The article "Risk management system and intelligent decision-making for prefabricated building project under deep learning modified teaching-learning-based optimization" was retracted in 2025. Reasons: compromised peer review; unreliable results or conclusions; concerns about the peer review; concerns about the article.

# Risk management system and intelligent decision-making for prefabricated building project under deep learning modified teaching-learning-based optimization

**DOI:** 10.1371/journal.pone.0235980

**Published:** 2020-07-17

**Authors:** Huazan Liu, Yukang He, Qichao Hu, Jianfei Guo, Lan Luo

**Affiliations:** School of Civil Engineering and Architecture, Nanchang University, Nanchang, PR China; University College London, UNITED KINGDOM

## Abstract

This study establishes a model of prefabricated building project risk management system based on the Modified Teaching-Learning-Based-Optimization (MTLBO) algorithm and a prediction model of deep learning multilayer feedforward neural network (Backpropagation, BP neural network) to improve the requirements of risk management during the construction of large prefabricated building projects. First, we introduced the BP neural network algorithm based on deep learning. Second, the traditional Teaching-Learning-Based Optimization (TLBO) algorithm was modified by using information entropy, and the modified algorithm was simulated and tested in five test functions. Then, based on the BP neural network and MTLBO algorithm, we established the MTLBO-BP neural network prediction model and tested its performance. Finally, based on the MTLBO-BP neural network prediction model, MATLAB software was used to establish an intelligent model of the risk management system during the construction of prefabricated building projects, and the example verification was performed. In addition, the MTLBO algorithm was verified by test function simulation and established that global searchability is stronger than the TLBO algorithm. Of note, it is not easy to fall into a local optimum. The test results of the MTLBO-BP neural network prediction model revealed that the prediction model converges faster and exerts a better prediction effect. The example verification of the intelligent model of the risk management system during the construction of prefabricated building projects established in this study revealed that the algorithm proposed is more accurate in the reliability and cost prediction of the risk management of prefabricated building projects. Moreover, the algorithm proposed provides theoretical support for intelligent management and decision-making of prefabricated building projects. Overall, this study validates that this algorithm is essential for construction project management, decision-making, and quality assurance.

## 1. Introduction

The construction industry is a crucial pillar industry in China and plays an irreplaceable role in promoting the development of the national economy and national urbanization. However, some hidden safety hazards and environmental problems have become increasingly prominent with the massive development of the construction industry [1]. Statistically, during 2010–2017, the total number of safety production accidents in municipal engineering in China was 4521 [2]. Among them, 209 were major accidents, with over 5000 deaths. Thus, the safety problem in the construction industry is critical [3]. In addition, the total energy consumption of China’s construction industry in 2016 accounted for >20% of that of the country, and the accompanying emissions also accounted for a large proportion. Thus, the construction industry is also encountering a growing number of environmental problems [4]. Based on the increasingly prominent safety and environmental problems of the traditional construction industry, the government has formulated a series of related policies to endorse the development of new construction industries. Indeed, there are many policies on dynamically promoting the development of prefabricated buildings; these policies not only provide incentives and subsidies to units implementing prefabricated building projects but also strongly support the improvement and standardization of prefabricated building technologies and standards [5]. Prefabricated building implies the building assembled with prefabricated components on the construction site, which is characterized by convenient construction, low cost, and short construction period. Compared with traditional cast-in-situ buildings, the use of prefabricated buildings offers higher advantages in terms of environmental, economic, and social benefits [6]. Thus, at the current stage of the construction industry, it is crucial for the development of prefabricated buildings to address the hidden safety hazards and prevent or minimize human casualties during the construction process. The development of prefabricated buildings in developed countries started earlier, and research on the construction risk of prefabricated buildings also preceded China. Maryam et al. [7] investigated the safety hazards of 125 prefabricated building construction sites by analyzing the data of occupational safety accident investigation in the United States; they identified the factors causing the injury and the potential factors, including the instability of the connection between components, resulting in the fall from high altitude [7]. A growing number of scholars in China have explored the safety aspect of prefabricated building construction, including safety management measures and risk assessment methods. Lin et al. [8] developed a process of integrating various stakeholders, information, and data through the building information model of information technology. Combining prefabricated procedures and the most advanced construction technology platform, the model was used to supervise the construction status; notably, it can improve the success rate of daily operations and decision-making in the full life-cycle management of the building, thereby reducing key schedule risks and ensuring timely project delivery [8].

With the rapid advancement of artificial intelligence, Artificial Neural Network (ANN) based on deep learning has been extensively used in computer vision, speech recognition, natural language processing, audio recognition, and bioinformatics. Currently, the most extensively used in ANN is the BP neural network. Larson et al. [9] examined the performance of deep learning neural network models in assessing the pediatric hand X-ray bone maturity [10]. Andrea et al. [11] applied deep neural networks to unregistered multitemporal images to attain multi-image super-resolution [12]. The TLBO algorithm is a swarm intelligence optimization algorithm proposed by Indian scholar Rao in 2011 [13]; the advantage of this algorithm is that the parameter setting structure is simple and easy to understand, the solution speed is fast, and it has strong convergence ability and global searchability. In addition, the algorithm has been applied to optimization design in various fields such as mechanical design, steel frame optimization design, and optimization of mechanical processing problems [14]. However, research of the Teaching-Learning-Based Optimization (TLBO) algorithm in prefabricated building projects remains limited. Furthermore, the basic TLBO has disadvantages of being easy to fall into local optimum and poor global search performance.

Thus, based on the TLBO, deep learning neural network and information entropy are used in this study to improve its algorithm. In addition, the risk management and control system model of the intelligent prefabricated building is established. We use Modified Teaching-Learning-Based Optimization (MTLBO) to optimize the model. Furthermore, different control strategies are proposed to examine the reliability of prefabricated residential construction system to enhance the quality and safety of prefabricated buildings and promote the green development of the construction industry.

## 2. Methods

### 2.1 BP neural network algorithm based on deep learning

Deep learning-based ANN is a mathematical model derived by imitating the nervous system of the human brain to process complex information with the central nervous network of the human brain as a principle; it has strong learning ability, self-adaptive ability, and nonlinear function approximation ability, as well as its fault-tolerance rate is high. The simulation model can be established for the recognition, prediction, and fuzzy control of binary images. The BP neural network is a type of ANN, which belongs to the multilayer feedforward neural network of backpropagation; it comprises a three-layer structure, including an input layer, implicit layer, and output layer. Fig 1 shows the schematic diagram of the BP neural network structure [9].

**Fig 1:** BP neural network structure diagram.

Fig 1 shows that each layer of the BP neural network comprises *n* neurons, and the layers are interconnected. However, the neurons in the layer are not connected. The algorithm includes two processes—error backpropagation and forward propagation of information. Fig 2 shows the specific process of the BP neural network algorithm.

**Fig 2:** BP neural network algorithm process.

In the forward propagation process, the input object was divided into *n* input vectors; *w* denotes the weight coefficient, while *b* denotes the bias vector. We performed a linear operation on the input vector *x*. The operation function is shown below:

$$z_{i}=\sum_{i}w_{i}{}_{n}•x_{n}+b_{i}$$ (1)

where *z*_*i*_ is the output of the *i*th layer neuron; *w*_*in*_ denotes the weight coefficient of the *n*th neuron; and *b* is the bias vector. The function calculates layer by layer from the input layer until the result is output. The BP neural network often uses the sigmoid function as the activation function of the inner layer of neurons to enhance the algorithm’s ability to express the model. The expression of the sigmoid function g(z_i_) is as follows:

$$g\left(z_{i}\right)=\frac{1}{1+e^{-z_{i}}}$$ (2)

The domain of the function provided above is all real number sets, and the range is [0,1]. After the last hidden layer outputs the result, the cross-entropy loss function evaluates the loss of the output; it is used to predict the gap between the output and the actual value, as well as measure the predictive ability of the model [11]. The loss function can be expressed as follows:

$$\text{loss}=-\frac{1}{n}\sum_{x}[y\;ln\;g\left(z_{i}\right)+\left(1-y)\;ln\;(1-g\left(z_{i}\right)\right)]$$ (3)

where *y* is the actual output value. When the loss value is exceptionally high, the parameter update is faster; else, the parameter update is slower.

During error backpropagation, the loss function gradient is back-propagated from the output layer to the hidden layer, and the loss value is distributed to the neurons in each layer. Through continuous iteration, the parameters between the layers are updated to minimize the error between the actual output value and the expected output value. Thus, the weight and threshold corresponding to the minimum error are identified, and the robustness of the BP neural network is enhanced. Based on the loss function gradient descent method, along the process of backpropagation, the gradient descent is the largest.

$$w_{i+1}=w_{i}-lr•\nabla$$ (4)

$$\nabla =\frac{\partial \text{loss}}{\partial w}$$ (5)

where *w*_*i+*1_ implies the updated weight coefficient; *w*_*i*_ denotes the current weight coefficient; lr is the learning rate of the number of iterations; and ∇ is the loss function gradient.

### 2.2 MTLBO algorithm

Traditional teaching algorithms include an initialization class group, a teaching stage, and a learning stage. In the initial stage, no difference exists between students. By learning from teachers during the teaching and learning stages, the performance of different students is unstable. As the number of iterations increases, the degree of student dispersion increases, and it is easy to fall into a local optimum. In the evaluation of high-dimensional problems, global searchability becomes weak [15]. Thus, under traditional TLBO, we proposed a method based on information entropy to modify TLBO, to overcome the limitations of TLBO easily falling into a local optimum, and enhance global searchability.

The MTLBO algorithm process is as follows:

(1) Initialization class: A class is randomly selected in the search space, and each student is represented, as shown below:
  $$X^{j}=(x_{1}^{j},x_{2}^{j},\ldots ,x_{d}^{j})\;(j=1,2,\ldots ,\text{NP})$$ (6)
  where *j* denotes the student number, and *d* is the number of subjects.
(2) Teaching stage: Teachers teach according to the differences between themselves and students. The teaching process is as follows:
  $$X_{\text{new}}^{i}=X_{\text{old}}^{i}+\text{difference}$$ (7)
  $$\text{Difference}=r_{i}\times \left(X_{\text{teacher}}-TF_{i}\times \text{mean}\right)$$ (8)
  where $X_{new}^{i}$ and $X_{old}^{i}$ denote the students’ values before and after learning; “Difference” represents the differences between teachers and students; *r*_*i*_ denotes the teaching step and is defined as rand (0,1); TF is the teaching factor, usually defined as 1 or 2; and “mean” represents the students’ average performance. Then,
  $$TF_{i}=\text{round}\left(1+\text{rand}\left(0,1\right)\right)$$ (9)
  $$\text{mean}=\frac{1}{\text{NP}}\sum_{i=1}^{\text{NP}}X^{i}$$ (10)

In the process of students learning from the best individual teachers, the learning levels are random and diverse. Thus, students’ performance while learning from teachers is uncertain. Of note, information entropy is used to represent the degree of dispersion of student performance. The lower the entropy value, the higher the degree of dispersion. At this time, the teaching factor (TF) should be high to hasten the search speed of the algorithm; however, it would reduce searchability. When the entropy value is high and the degree of dispersion is small, the distribution of student performance differences is more regular. Thus, the TF should be small to make the search accuracy more subtle; however, meanwhile, the search speed would be reduced to a certain extent. The performance probability distribution of the *j*th student in subject *i* is defined as follows:

$$P\left(x_{i}^{j}\right)=\frac{x_{i}^{j}}{\sum_{j=1}^{\text{NP}}x_{i}^{j}}$$ (11)

Then, the information entropy of the subject *i* is as follows:

$$S_{i}=-\sum_{j=1}^{\text{NP}}P\left(x_{i}^{j}\right)\text{log}P\left(x_{i}^{j}\right)$$ (12)

After introducing information entropy, the improved teaching factor is presented as follows:

$$TF_{i}=TF_{\text{max}}-(\frac{TF_{\text{max}}-TF_{\text{min}}}{S_{\text{max}}})*S_{i}$$ (13)

Information entropy can be obtained according to Eqs (11) and (12). The new individuals after the completion of the teaching stage could be obtained according to Eqs (7)–(10). If the new solution is better than the original solution, the new solution is chosen; else, the student position will not be updated.

(3) Learning stage. Each student *X*^*i*^ randomly selects a learning object *X*^*j*^ in the class and learns through the difference between the two. The learning process is shown as follows:
  $$X_{\text{new}}^{j}=\{\begin{array}{l} X_{\text{old}}^{j}+r\times \left(X^{j}-X^{r}\right),f(X^{r})<f(X^{j})\\ X_{\text{old}}^{j}+r\times \left(X^{r}-X^{j}\right),f(X^{r})>f(X^{j}) \end{array}$$ (14)
  where *r* is the learning step, and the value range is [0, 1]. The update operation is shown below.
  $$If\;f\left(X_{\text{new}}^{i}\right)>f\left(X_{\text{old}}^{i}\right),X_{\text{new}}^{i}=X_{\text{old}}^{i}$$ (15)

If the termination condition is fulfilled, the iterative operation ends; else, the operation is repeated from step (2). Based on the algorithm steps listed above, Fig 3 shows the specific operation process of MTLBO.

**Fig 3:** MTLBO algorithm process.

According to Fig 3, the specific process of the MTLBO algorithm is as follows: (i) a specific number of students are randomly generated according to the specific optimization problem. Then, the class and algorithm parameters are initialized. (ii) The fitness of each individual in the class is evaluated, and the individual with the best fitness is selected as the teacher. (iii) The information entropy is calculated according to Eqs (11) and (12). (iv) Based on the information entropy, the teaching stage is started, and the new solution is compared with the old solution to update the student position. (v) If the new solution is better than the old solution, the new solution is selected as the new class individual, and the learning stage is started. (vi) The learning stage is implemented according to Eqs (14) and (15), enabling students to learn from each other, or according to their experience. (vii) If a student reaches a higher fitness level through learning, the position is updated. Moreover, the learning experience is updated according to Eq (8). (viii) Steps (2)–(7) are repeated until the termination condition is fulfilled.

### 2.3 MTLBO algorithm simulation test

We selected five functions with local optimal characteristics to validate the efficacy of the MTLBO algorithm in this study. Using MATLAB, the five functions were simulated and tested. Then, the test results of the MTLBO algorithm were compared with the traditional TLBO algorithm. The five test functions set the same parameters: the number of populations (NP) = 15; the maximum number of iterations (itermax) = 500; the teaching factor (TF_max_) = 2; TF_min_ = 1; *D* = 30. Of note, the two algorithms were operated independently 30 times, obtaining the average deviation and standard deviation of each algorithm for each test function. The average deviation is the average value of the optimal value obtained by multiple iterations of the algorithm, which depicts the accuracy of the algorithm’s solution. In addition, the robustness of the algorithm was reflected by the standard deviation. Table 1 presents the dimension, name, variable range, and exact value of each test function. The optimal value can judge global searchability of the algorithm. Through the dimension of each test function, the scope of the name variable, and the exact value, we observed that the five functions have local optimal characteristics, which could be used to determine global searchability of the TLBO and MTLBO algorithms [16].

**Table 1:** Test functions.

Function expression	Dimension	Function name	Variable range	Optimal value
$f_{1}=\sum_{i=1}^{n}x_{i}^{2}$	30	Sphere	[−100,100]	0
$f_{2}=\sum_{i=1}^{n}\frac{x_{i}^{2}}{4000}-\prod_{i=1}^{n}\text{cos}(\frac{x_{i}}{\sqrt{i}})+1$	30	Griewank	[−600,600]	0
$f_{3}=\sum_{i=1}^{n}(x_{i}^{2}-10\text{cos}(2\pi x_{i})+10)$	30	Rastrigin	[−5.12,5.12]	0
$f_{4}=\sum_{i=1}^{n}ix_{i}^{2}$	30	Sum square	[−10,10]	0
$f_{5}=\sum_{i=1}^{n}(\sum_{j=1}^{i}x_{j}{)}^{2}$	30	Quadric	[−10,10]	0

### 2.4 Establishment of the MTLBO-BP neural network prediction model

The randomness of the initialization of the BP neural network could create the problem of uncertain final output results or poor convergence. Thus, we optimized the MTLBO algorithm based on the deep learning BP neural network. In addition, we used the three-layer structure of the BP neural network to encode the individual students of the MTLBO algorithm—*X*_*i*_ = (*w*_1_, *B*_1_, *w*_2_, *B*_2_ …, *w*_*n*_, *B*_*n*_); *w*_1_ denotes the weight coefficient, and *B*_1_ is the threshold vector. Then, the optimized objective function of the MTLBO algorithm was the mean square error output by the BP neural network. The smaller the mean square error, the better the students’ fitness. Based on the optimized objective function, students with optimal fitness were obtained and decoded. Then, the initial weight and threshold of the BP neural network were set according to the optimal individuals obtained by the MTLBO algorithm; this way, the global optimal solution could be obtained by establishing the MTLBO-BP prediction model. Fig 4 shows the specific MTLBO-BP prediction model process.

**Fig 4:** MTLBO-BP prediction model process.

We compared and analyzed the standard BP neural network model and the MTLBO-BP neural network prediction model to test the efficacy of the MTLBO-BP prediction model established in this study. The two prediction models were set with the same parameters—the maximum number of iterations, 300; the population initialization range, [–1, 1]; the number of hidden layer nodes, *m*; the individual dimension, *d*; and the dataset of the number of population, NP. We selected four sets of typical real test data from the dataset, as shown in Table 2. Accordingly, the two prediction models mentioned above were tested. Of note, the dataset was derived from the UCI dataset; it belongs to real test data, which is more convincing to validate the efficacy of the two prediction models.

**Table 2:** Test data and parameters.

Dataset	Dimensions	Number of training samples	Number of test samples	*m*	*d*	NP
Parkinsons	18	2100	425	3	25	35
Wine Quality	13	1300	480	3	36	30
Concrete Strength	10	600	208	2	67	25
Airfoil Self-Noise	7	900	370	1	84	15

### 2.5 Design of the model for the safety risk management system of prefabricated building construction

Based on the MTLBO-BP prediction model, we designed the model of the safety risk optimization system of the prefabricated building. The installation process of various prefabricated components was used as the basic construction process, and each basic construction process was used as a subsystem to represent various subjects of the MTLBO algorithm. For each system [17], the various subjects’ performance of the optimal individual obtained after the entire class was optimized, which could represent the best choice of each subsystem. The BP neural network parameters were set according to the optimal individual, and MATLAB was used to build an intelligent model for safety risk optimization of prefabricated buildings, which could predict and analyze the reliability of construction projects. Based on the results, different strategies were adopted to provide new ideas for the management of prefabricated building projects.

Finally, we selected a prefabricated building project in a certain city as a sample to validate the model and analyzed the results by numerical simulation methods. The main structure of the project selected was a shear wall structure. The inner wall panels, outer wall panels, stairs, and balconies of the main structural part were all assembled using prefabricated components. In addition, the structural floor and stairs were made of laminated boards. The bathroom adopted an integral prefabricated structure, and air-conditioning panels, nodes, and joints were cast on site. Table 3 presents the basic information of each subsystem.

**Table 3:** Basic information of each subsystem.

Serial number	Subsystem name	Time of duration/h	Cost/Yuan	Engineering quantity	
				Unit	Quantity
1	Earthwork	11	120	m^3^	3823
2	Foundation engineering	7	3270	m^3^	1708
3	Column installation project	45	9278	m^3^	823
4	Beam installation project	144	9224	m^3^	1109
5	Plate installation project	43	10,476	m^3^	102
6	Reinforcement binding and pipeline Embedment	25	3827	m^3^	548
7	Concrete pouring	25	4935	m^3^	276
8	Wall panel installation project	38	15,108	m^3^	2501
9	Stair installation project	41	12,289	m^3^	51
10	Installation of superimposed balcony slab	37	11,956	m^3^	76
11	Integral bathroom installation	20	8803	Number	120
12	Supporting protection system	44	6165	Number	1276
13	Completion acceptance	5	14,615	Number	1

We assumed that the number of prefabricated components purchased for the project was sufficient, as well as the transportation, storage, and fixing of materials could fulfill the conditions for the smooth progress of the project. Through MATLAB, the MTLBO-BP prediction calculation model was operated to set the initial parameters—the number of population (*N* = 100); the maximum teaching factor (TF_max_ = 2); the minimum (TF_min_ = 1); and the number of iterations was 500 times. Based on the best results, the best allocation scheme was obtained. Furthermore, the results obtained by the algorithm were compared with those calculated by the genetic algorithm.

## 3. Results and discussion

### 3.1 MTLBO algorithm simulation results

We selected five functions with local optimal characteristics to validate the efficacy of the MTLBO algorithm. Based on the test results of the two algorithms, the average deviation and standard deviation data of each function were obtained, as shown in Table 4.

**Table 4:** MTLBO algorithm simulation results.

Test function	TLBO		MTLBO	
	Average deviation	Standard deviation	Average deviation	Standard deviation
f_1_	1.48e–820	2.60e–790	0	0
f_2_	0	0	0	0
f_3_	2.12e–152	9.70e–150	0	0
f_4_	9.68e–2	4.98e–2	9.53e–2	1.01e–2
f_5_	9.20e–41	1.79e–40	0	0

Based on the test results of the average deviation and standard deviation of the MTLBO algorithm and the basic TLBO algorithm in the five test functions (Table 4), we observed that the MTLBO algorithm achieved high accuracy in the operation of these five high-dimensional complex functions, especially the global optimal solution was obtained in the functions f1, f2, f3, and f5. In addition, the basic TLBO algorithm only reached the global optimal solution in function f2, and the rest fell into the local optimal solution. Thus, the MTLBO algorithm in this paper has strong searchability in solving large-scale complex optimization problems. Based on the simulation test results, we obtained the optimal convergence curves of the two algorithms in the Griewank and Rastrigin functions, as shown in Figs 5 and 6.

**Fig 5:** Convergence curves of the two algorithms in the Griewank function.

**Fig 6:** Convergence curves of the two algorithms in the Rastrigin function.

Based on the premise that both the TLBO and MTLBO algorithms could reach the global optimal solution, f_2_: Griewank function was selected. One of the remaining four random functions, f_3_: Rastrigin function, was used to compare the phenomenon that the MTLBO algorithm reached the global optimal solution, and the TLBO algorithm reached the local optimum. As shown in Figs 5 and 6, the MTLBO algorithm converges to the optimal value in the Griewank function when the number of iterations function is 40. In addition, the TLBO algorithm converges to the optimal value in the Griewank function when the number of iterations is nearly 120. Moreover, the MTLBO algorithm converges to the optimal value in the Rastrigin function when the number of iterations is 8. The TLBO algorithm converges to the optimal value in the Rastrigin function when the number of iterations is approximately 50. Notably, the MTLBO algorithm tends to converge to the global optimal solution at a faster speed, whereas the TLBO algorithm has a slower convergence speed or falls into a local optimum. From the simulation test results provided above, it can be deduced that the convergence speed of the MTLBO algorithm has been significantly improved, and it is easy to jump out of the local optimum to achieve the expected effect. Hence, the proposed MTLBO algorithm has strong robustness and stability.

### 3.2 Test results of the MTLBO-BP neural network prediction model

The test data and parameters listed in Table 2 were used to test the MTLBO-BP neural network prediction model. Fig 7 shows the prediction percentage errors of the two neural network prediction models, and the average training time shown in Fig 8 can be obtained.

**Fig 7:** Prediction percentage error.

**Fig 8:** Average training time.

According to Fig 7, for the actual dataset presented in Table 2, the optimal weight and threshold of the BP neural network are often not at the origin. The MTLBO algorithm improves the initial weight and threshold of the deep learning BP neural network algorithm. Thus, compared with the BP neural network model, the average prediction relative percentage error of the MTLBO-BP neural network model has been decreased by 9.43%, 7.32%, 3.82%, and 1.90% on the four datasets. As shown in Fig 8, compared with the BP neural network model, the training time of the MTLBO-BP neural network model on the four datasets has been decreased by 23.8%, 25.7%, 21.7%, and 45.0%, respectively. The comparison of the test results of the two prediction models establishes that the MTLBO-BP neural network model has a better prediction effect. Moreover, the MTLBO-BP model exerts a certain effect on the improvement of the initial weights and thresholds of the BP neural network algorithm. Furthermore, it improves the limitations of the basic TLBO, which can easily fall into the local optimum and has poor global search performance.

### 3.3 Optimization results of the prefabricated building safety risk system model

We compared the calculated results with the results obtained by the genetic algorithm. Table 5 shows the reliability results of the construction system.

**Table 5:** Comparison of reliability optimization results of construction projects with two different algorithms.

Construction project	MTLBO-Neural network		GA	
	Reliability	Cost	Reliability	Cost
1	0.831	120	0.821	122
2	0.719	3270	0.728	3274
3	0.652	9278	0.649	9279
4	0.773	9224	0.778	9226
5	0.824	10,476	0.822	10,479
6	0.541	3827	0.503	3828
7	0.694	4935	0.679	4937
8	0.683	15,108	0.684	15,111
9	0.849	12,289	0.847	12,292
10	0.732	11,956	0.721	11,957
11	0.749	8803	0.746	8805
12	0.811	6165	0.806	6168
13	0.673	14,615	0.667	14,617

Table 5 shows that the optimization results of each subsystem based on the MTLBO-BP prediction model algorithm are better than those obtained by the genetic algorithm. From the cost obtained by the reliability of the construction system, the project cost based on the MTLBO-BP prediction model algorithm is low. Thus, the proposed method has reliability and superiority. Hence, this study demonstrates that the MTLBO-BP prediction model based on deep learning can be applied in the prefabricated building project management. According to the intelligent prediction model, different strategies could be adopted to provide a theoretical basis for the management of large-scale prefabricated building projects.

## 4. Conclusions

This study establishes the risk intelligent management system model for prefabricated construction engineering projects by combining the BP neural network algorithm based on deep learning and the MTLBO algorithm based on information entropy. Each subsystem of the construction project is optimized to determine the best project allocation scheme. This study demonstrates that the MTLBO-BP neural network prediction model optimized by the MTLBO algorithm has better prediction performance. In addition, the intelligent model of the risk management system for prefabricated building projects based on the algorithm has a faster convergence speed and a more accurate solution to the problem of reliability and cost allocation of engineering projects. Our proposed model can provide theoretical support for the management and decision-making of prefabricated building projects. Thus, the proposed algorithm is immensely significant for construction project management, decision-making, and quality assurance. However, there exist some limitations. In terms of model establishment and algorithm operation, the modified algorithm could solve the general-scale prefabricated construction process. However, more large-scale construction projects would increase in the future. Hence, further research is warranted in terms of algorithm improvement and rational construction of models.

## Supporting information

S1 Data (XLS)

S1 File (DOC)
